The article "Clinical Effect of Clarithromycin Combined with Tinidazole on Helicobacter pylori-Related Gastritis and Its Influence on COX-2 Expression" was retracted in 2024. Reasons: signs of a paper mill; suspected computer-generated content; unreliable results or conclusions; concerns about the data.

# Clinical Effect of Clarithromycin Combined with Tinidazole on Helicobacter pylori-Related Gastritis and Its Influence on COX-2 Expression

**DOI:** 10.1155/2021/4171019

**Published:** 2021-11-30

**Authors:** Chenxi He, Fanting Kong, Xinying Zhu, Fanlei Kong, Wei Zhao, Yanling Liu, Kuixiang Wang

**Affiliations:** ^1^Department of Gastroenterology, Xingtai People's Hospital, Xingtai, 054000 Hebei Province, China; ^2^Department of Breast Surgery, Xingtai People's Hospital, Xingtai, 054000 Hebei Province, China; ^3^Department of Gastroenterology, The Third Affiliated Hospital of Hebei Medical University, Shijiazhuang, 050000 Hebei Province, China; ^4^Department of Orthopedics, Xingtai People's Hospital, Xingtai, 054000 Hebei Province, China

## Abstract

Studies have shown that COX-2 expression is upregulated in gastric cancer (GC) as well as in precancerous lesions and in Helicobacter pylori-induced inflammation, suggesting that cyclooxygenase-2 (COX-2) may play an important role in gastric carcinogenesis. We attempted to investigate the role of clarithromycin with tinidazole on Helicobacter pylori-related gastritis from the aspects of clinical effect and COX-2 expression. From January 2016 to January 2019, 130 patients with Helicobacter pylori-related chronic gastritis were collected and grouped into the observation group (OG) and the control group (CG). Altogether, 80 patients in the OG were treated with clarithromycin with tinidazole, while 50 patients in the CG were treated with amoxicillin with metronidazole. Clinical symptom improvement time, content of COX-2 and B cell lymphoma-2 (BCL-2), content of inflammatory factors interleukin-1 (IL-1), IL-4, and C-reactive protein (CRP), expression level of nutritional indicators serum albumin (ALB), realbumin (PA), and transferrin (TF), clearance of Helicobacter pylori, total effective rate, and incidence of adverse reactions were detected. Compared with the CG, the OG had shorter clinical symptom improvement time, lower COX-2 and Bcl-2, lower expression of inflammatory factors IL-1, IL-4, and CRP, higher expression of nutritional indicators ALB, TF, and PA, higher clearance rate of Helicobacter pylori, higher total effective rate, and lower incidence of adverse reactions. Clarithromycin combined with tinidazole can effectively improve the clinical effect of Helicobacter pylori-related gastritis and reduce the expression level of COX-2.

## 1. Introduction

Helicobacter pylori, a gram-negative bacterium, exists in the stomach, and its infection rate is as high as 90% all over the world, and about 20%-30% of infected people will undergo some kinds of diseases, including peptic ulcer, gastric carcinoma, or mucosa-related lymphoid tissue lymphoma [1–3]. In both developed and developing countries, Helicobacter pylori infection is closely related to the cross-living environment and hereditary susceptibility [4, 5]. The gastritis induced by it is chronic and can develop into atrophic gastritis, intestinal metaplasia, and dysplasia. At the same time, cyclooxygenase-2 (COX-2), an important factor in Helicobacter pylori-associated gastritis, angiogenesis, and inhibition of apoptosis in gastric carcinoma are evidently related to infiltration [6–8]. Recently, studies have shown that COX-2 expression is upregulated in GC as well as in precancerous lesions and in Helicobacter pylori-induced inflammation, suggesting that COX-2 may play an important role in gastric carcinogenesis [8, 9]. Chronic atrophic gastritis caused by Helicobacter pylori activates synthesis of growth factors and cytokines leading to elevated COX-2 expression [6, 8]. Studies in vitro find that Helicobacter pylori was correlated with an upregulation of the expression of COX-2 mRNA/protein 2 in gastric cancer (GC) cell line. Therefore, the relatively early role of COX-2 in gastric carcinogenesis makes it an attractive target for cancer chemoprevention [6–11].

The article "Clinical Effect of Clarithromycin Combined with Tinidazole on Helicobacter pylori-Related Gastritis and Its Influence on COX-2 Expression" was retracted in 2024. Reasons: signs of a paper mill; suspected computer-generated content; unreliable results or conclusions; concerns about the data.

Clarithromycin interacts with peptidyl transferases of partial RNA of bacteria, which can effectively inhibit the activity of bacterial ribosomes and hinder the synthesis of proteins [12]. But the problem is that bacterial RNA is easy to mutate, which will lead to bacterial resistance to clarithromycin [13]. Tinidazole is a relatively new nitroimidazole derivative, which has strong antibacterial activity, good pharmacokinetic characteristics, and less side effects and is a good antibacterial drug [13]. Because of their good antibacterial properties, these two drugs are often used alone or in combination in various bacterial diseases [14–16]. In this study, we intended to explore the effects of clarithromycin and tinidazole on Helicobacter pylori and inflammation elimination. However, the effect of the combined use of the two drugs in Helicobacter pylori-related gastritis is still unclear. In this study, we studied the combination of two drugs and its influence on COX-2.

## 2. Method

### 2.1. Data

From January 2016 to January 2019, 130 Helicobacter pylori-related chronic gastritis patients were collected and grouped into the observation group (OG) and the control group (CG). The OG consisted of 43 men and 37 women, aged 32-57 years with an average age of 42.13 ± 1.21 years. The CG consisted of 28 men and 22 women, aged 31-58 years with an average age of 41.87 ± 1.53 years. There was no evident difference in general data between the CG and the OG (*p* > 0.05), but it was comparable. This research has been approved by the ethics committee. The family members and the patients have signed the informed consent form.

The article "Clinical Effect of Clarithromycin Combined with Tinidazole on Helicobacter pylori-Related Gastritis and Its Influence on COX-2 Expression" was retracted in 2024. Reasons: signs of a paper mill; suspected computer-generated content; unreliable results or conclusions; concerns about the data.

Inclusion criteria include patients have abdominal discomfort, burning pain, fullness, pantothenic acid, belching, and other symptoms; patients were confirmed as superficial gastritis or atrophic gastritis by gastroscopy; after 13C breath test, bacterial culture, and urease test, the results were positive, and there was direct evidence of Helicobacter pylori infection. Exclusion criteria include patients with severe hepatic and renal insufficiency and tumors; patients have contraindications to the drugs used in this study; patients were unconscious or suffered from mental illness; patients had communication barriers; patients did not cooperate with clinical treatment.

### 2.2. Methods

Patients in the CG were given amoxicillin combined with metronidazole for Helicobacter pylori-related gastritis, in which amoxicillin [manufacturer: Shanghai Haihong Group Chaohu C-Dragon Pharmaceutical Co., Ltd., SFDA Approval No. H34023991; specification: 125 mg (calculated by C16H199N3O5S)] was taken with warm water, three times a day, and each time was applied according to the patient's body mass, 5 mg/kg. Combined use of metronidazole (manufacturer: Fujian Yoshida Huamin Antibiotics Co., Ltd., SFDA Approval No. H35020323; specification: 200 mg) was applied with warm water, 3 times a day, 7 mg/kg. Fourteen days indicated a course, and a total of two courses were performed.

Patients in the OG were treated with clarithromycin and tinidazole, among which clarithromycin (manufacturer: Hainan Hewlett-Packard Medical Biotechnology Co., Ltd., SFDA Approval No. H20040649; specification: 125 mg) was taken with warm water, 3 times a day, and each amount was taken according to the patient's body mass, 0.5 mg/kg. At the same time, tinidazole was used in combination (manufacturer: Guangzhou Baiyunshan Pharmaceutical Holdings Co., Ltd., Baiyunshan Pharmaceutical General Factory, SFDA Approval No. H44021435; specification: 500 mg) and taken with warm water once a day, and each time was measured according to the patient's body mass, 15 mg/kg. Fourteen days indicated a course, and a total of two courses were performed.

### 2.3. Detection Indicators

#### 2.3.1. Improvement Time of Clinical Symptoms

The improvement of clinical symptoms was observed and compared, including belch improvement time, epigastric pain improvement time, acid reflux improvement time, and abdominal distension improvement time.

#### 2.3.2. Content of Cox-2 and Bcl-2

Before treatment and 14 days and 30 days after treatment, the mRNA contents of COX-2 and Bcl-2 were detected and compared. Before treatment and 14 days and 30 days after treatment, 3 ml of fasting venous blood was taken from a vacuum nonanticoagulation tube, placed at room temperature for 30 min, and centrifuged at 1500 × *g* at 4°C for 10 min. Then, the upper serum was taken and detected by qPCR. First, total RNA in the blood was extracted: about 50 mg of plasma was moved into a 1.5 ml RNAse-free centrifuge tube, and 0.5 ml of TRIzol was added. After shaking, 0.5 ml of TRIzol was put in, and then, the whole process was lasted for about 30 minutes. A total of 200 *μ*l chloroform was added to every 1 ml TRIzol, which was quickly shaken and mixed for 30 s, then placed on ice for 5 min, and then centrifuged at 1500 × *g* at 4°C for 10 min. A pipette was applied to transfer about 400-600 *μ*l of supernatant to a new centrifuge tube; then, 500 *μ*l/1 ml TRIzol isopropanol was added, covered, mixed upside down repeatedly, then placed for 10 min, put into a centrifuge, and centrifuged at 1500 × *g* at 4°C for 10 min. The supernatant was discarded, isopropyl alcohol was absorbed, and 1 ml of 75% ethanol was added and mixed well. It was centrifuged at 1500 × *g* at 4°C for 10 min, and RNA was washed. The supernatant was discarded and dried naturally for 5-10 min, and 20 *μ*l DEPC water was applied to dissolve the total RNA. Then, qPCR was carried out in ABI7500 fluorescence quantitative PCR instrument in the USA, and the steps were as follows: 95°C for 5 min, 95°C for 15 s, and 60°C for 30 s, for a total of 40 cycles, and 60~95°C. Compared with internal reference, Bcl-2/GAPDH and COX-2/GAPDH were obtained. The ratio represents the relative expression level (Table 1).

The article "Clinical Effect of Clarithromycin Combined with Tinidazole on Helicobacter pylori-Related Gastritis and Its Influence on COX-2 Expression" was retracted in 2024. Reasons: signs of a paper mill; suspected computer-generated content; unreliable results or conclusions; concerns about the data.

Before treatment and 14 days and 30 days after treatment, COX-2 and Bcl-2 were detected and compared. Cox-2 and Bcl-2 protein, Bcl-2/GAPDH, and COX-2/GAPDH in serum of the CG and the OG were tested by Western blot. The ratio represents the relative expression level.

#### 2.3.3. Level of Inflammatory Factors

Before treatment and 14 days and 30 days after treatment, COX-2 and Bcl-2 in the blood of the two groups were detected and compared. Interleukin-1 (IL-1), interleukin-4 (IL-4), and serum C-reactive protein (CRP) were compared by ELISA.

#### 2.3.4. Nutritional Indicators

Before treatment and 14 days and 30 days after treatment, the nutritional indexes in the blood of the CG and the OG were detected and compared. The nutritional indexes of the patients were detected by ELISA, and some plasma samples were collected to detect the serum albumin (ALB), prealbumin (PA), and transferrin (TF).

#### 2.3.5. Clearance of Helicobacter pylori

After treatment, the clearance of Helicobacter pylori was examined. The two groups were examined by gastroscopy, and Hp was detected by 14C-urea breath test. If the bacteriological examination results are negative after treatment, the patients who are reinfected by the same pathogenic bacteria are counted as the number of reinfected cases. If the results are positive for two consecutive times after treatment, it is counted as the number of uncleaned cases. If the results are negative for two consecutive times after treatment, it is counted as the number of clearance cases. After that, the bacterial clearance rate of the two groups of patients was calculated, bacterial clearance rate = (cleared cases/total cases) × 100%.

The article "Clinical Effect of Clarithromycin Combined with Tinidazole on Helicobacter pylori-Related Gastritis and Its Influence on COX-2 Expression" was retracted in 2024. Reasons: signs of a paper mill; suspected computer-generated content; unreliable results or conclusions; concerns about the data.

#### 2.3.6. Total Effective Rate

After treatment, the total effective rate of patients was counted. The criteria are as follows: symptoms such as fullness, loss of appetite, and stomachache disappeared after meals, and gastroscopy showed that the ulcer surface healed, which was cured; symptoms such as fullness, loss of appetite, and stomachache after meals were evidently improved, and gastroscopy showed that the ulcer surface was reduced by >80%, which was markedly effective; after dinner, symptoms such as fullness, loss of appetite, and stomachache were alleviated, and gastroscopy showed that the ulcer surface was reduced by 50%~80%, which was effective; symptoms and signs were not improved, and gastroscopy showed that the ulcer surface was reduced by <50%, which was ineffective. Total effective rate = [(effective cases + markedly effective cases + cured cases)/total cases] × 100%.

#### 2.3.7. Adverse Reactions

The total incidence of adverse reactions of the CG and the OG after treatment was analyzed. The related indicators were nausea, dizziness, and vomiting.

### 2.4. Statistical Methods

SPSS 22.0 was applied for comprehensive data statistical analysis, and the measurement data were represented as *X* ± *S* and tested by *t*-test. The counting data were represented as *X*^2^. When *p* < 0.05, the difference is obvious and has statistical significance.

## 3. Results

### 3.1. General Information

There was no evident difference in general information such as gender, average age, average course of disease, and average weight between the CG and the OG (*p* > 0.05). See Table 2 for details.

### 3.2. The Improvement Time of Clinical Symptoms in the OG Was Shorter Than That in the CG

The belch improvement time, epigastric pain improvement time, acid reflux improvement time, and abdominal distension improvement time in the OG were shorter than those in the CG (*p* < 0.05). See Figure 1 for details.

### 3.3. Cox-2 and Bcl-2 in the OG after Treatment Were Lower Than Those in the CG

There was no evident difference in COX-2, Bcl-2 mRNA, and protein levels between the CG and the OG before treatment (*p* > 0.05). The mRNA and protein levels of Cox-2 and Bcl-2 in the OG were lower than those in the CG after 14 days of treatment (*p* < 0.05), but there was no difference between the CG and the OG after 30 days of treatment (*p* > 0.05). See Figure 2 for details.

The article "Clinical Effect of Clarithromycin Combined with Tinidazole on Helicobacter pylori-Related Gastritis and Its Influence on COX-2 Expression" was retracted in 2024. Reasons: signs of a paper mill; suspected computer-generated content; unreliable results or conclusions; concerns about the data.

### 3.4. The Level of Inflammatory Factors in the OG after Treatment Was Lower Than That in the CG

Comparing IL-2, IL-4, and CRP before treatment and 14 d and 30 d after treatment, it was found that there was no evident difference in IL-1, IL-4, and CRP between the CG and the OG before treatment (*p* > 0.05), but after treatment for 14 d and 30 d, IL-1, IL-4, and CRP in the CG and the OG decreased evidently. See Figure 3 for details.

### 3.5. After Treatment, the Nutritional Indexes of the OG Were Higher Than Those of the CG

Comparing the levels of nutritional indexes before treatment and after 14 days and 30 days of treatment, it was found that there was no evident difference in ALB, Tf, and PA levels between the CG and the OG before treatment (*p* > 0.05), but after 14 days and 30 days of treatment, the levels of ALB, Tf, and PA in the OG were evidently higher than those in the CG (*p* > 0.05). See Figure 4 for details.

### 3.6. The Clearance of Helicobacter pylori in the OG Was Better Than That in the CG

The clearance rate of Helicobacter pylori in the OG was evidently higher than that in the CG (*p* < 0.05). See Table 3 for details.

### 3.7. The Total Effective Rate of the OG Was Higher Than That of the CG

The total effective rates of the CG and the OG were compared. The total effective rate of the OG was evidently higher than that of the CG (*p* < 0.05). See Table 4 for details.

### 3.8. The Incidence of Adverse Reactions in the OG Was Higher Than That in the CG

Comparing the incidence of adverse reactions between the CG and the OG, it was found that the incidence of adverse reactions in the OG was evidently lower than that in the CG (*p* < 0.05). See Table 5 for details.

## 4. Discussion

Nowadays, Helicobacter pylori is the leading cause of a series of stomach diseases [17, 18]. For the treatment of Helicobacter pylori-related gastritis, it is necessary to use a treatment method with good antibacterial effect. In this study, we studied the effect of clarithromycin and tinidazole on C gastritis. In the discussion, we will discuss the combination of these two drugs on patients from the aspects of Helicobacter pylori, COX-2, and inflammatory factors.

In this experiment, the clearance rate of Helicobacter pylori in the OG was higher than that in the CG. In superficial gastritis caused by Helicobacter pylori, lymphocytes, polymorphonuclear leukocytes, and macrophages in gastric mucosa will be infected. With the passage of time, gastric mucosa will undergo further loss of glandular cells, which will eventually deteriorate into atrophic gastritis. Helicobacter pylori does not usually interact directly with immune cells in the stomach, yet components of the bacterium can exert their effects on these cells, leading to modulation of host inflammation [6, 12, 19]. Indeed, studies in an Helicobacter pylori mouse infection model showed that Helicobacter pylori vacuolating cytotoxin A (VacA) targets gastric lamina propria myeloid cells, thereby suppressing interleukin-23 (IL-23) expression by dendritic cells and inducing IL-10 and transforming growth factor-*β* (TGF-*β*) expression in macrophages. It was suggested that Helicobacter pylori uses VacA to promote tolerogenesis in the host [19]. Helicobacter pylori bacterial factors can also upregulate proinflammatory responses in immune cells thus leading to an exacerbation of inflammation. An example of this is the uncharacterized Helicobacter pylori protein HP1173 whose secretion levels vary significantly among strains. Recombinant HP1173 (rHP1173) was able to bind to THP-1 monocyte-derived macrophages, resulting in the production of the proinflammatory cytokines, tumor necrosis factor (TNF), and IL-1*β*, as well as the C-X-C motif chemokine ligand 8 (CXCL8), in a dose- and time-dependent manner [19].

The article "Clinical Effect of Clarithromycin Combined with Tinidazole on Helicobacter pylori-Related Gastritis and Its Influence on COX-2 Expression" was retracted in 2024. Reasons: signs of a paper mill; suspected computer-generated content; unreliable results or conclusions; concerns about the data.

In our study, in view of the results of this experiment on inflammatory factors, the level of inflammatory factors in the OG decreased faster, indicating that clarithromycin combined with tinidazole is more effective in eliminating Helicobacter pylori, and better pathogen elimination can alleviate the inflammatory reaction caused by this bacterium. In some studies, it was found that amoxicillin and metronidazole have poor clearance effect on Helicobacter pylori, and it is easy to cause bacterial drug resistance when they are combined with metronidazole [20, 21]. Clarithromycin is a good drug, but it can easily cause bacterial resistance. Tinidazole has been proved to be effective in the treatment of Helicobacter pylori infection and can be used as the first-line treatment drug for eradication of Helicobacter pylori. Its combination with clarithromycin can reduce the drug resistance of Helicobacter pylori caused by clarithromycin [22]. To sum up, it can be proved that clarithromycin combined with tinidazole has a better cleaning effect on Helicobacter pylori, thus reducing the inflammatory reaction.

According to the results of COX-2 and Bcl-2 in the CG and the OG, the mRNA and protein levels of COX-2 and Bcl-2 in the OG were lower after operation. Cox-2 is highly induced by various inflammatory cytokines in the site where inflammation occurs. Therefore, when gastritis occurs, inflammatory cytokines rise, leading to an increase in their levels. Upregulating of Cox-2 can even stimulate cell division and angiogenesis, inhibit apoptosis, and lead to the occurrence of gastric carcinoma [23]. Bcl-2 is another factor caused by inflammatory factors, which plays a promoting role in the carcinogenesis mediated by Helicobacter pylori infection [24]. Therefore, combined with the previous clearance results, we found that Helicobacter pylori can cause severe inflammatory reaction in the stomach, with the increase of inflammatory factors, COX-2, Bcl-2, and other factors, and then induce carcinoma in the stomach. Clarithromycin combined with tinidazole has a better bacterial clearance effect, and its role in treating Helicobacter pylori is to clean up Helicobacter pylori which induced diseases and then reduce the inflammation, reduce inflammatory factors, and inhibit the increase of COX-2 and Bcl-2 levels caused by inflammatory factors, thus effectively alleviating various symptoms caused by stomach inflammation. Therefore, we can see that some clinical symptoms in the OG have a shorter improvement time. The decrease of adverse reactions in the OG may be that there are fewer inflammatory factors and the symptoms are relieved better, so the incidence of adverse reactions is greatly reduced.

The article "Clinical Effect of Clarithromycin Combined with Tinidazole on Helicobacter pylori-Related Gastritis and Its Influence on COX-2 Expression" was retracted in 2024. Reasons: signs of a paper mill; suspected computer-generated content; unreliable results or conclusions; concerns about the data.

There are still some shortcomings in this experiment. We failed to investigate the satisfaction and dissatisfaction of patients by questionnaire when they were discharged from hospital. In the future research, we will pay attention to the treatment methods. At the same time, we should pay more attention to molecular mechanisms and the relationship between gastric carcinoma induced by Helicobacter pylori and these drugs.

To sum up, clarithromycin combined with tinidazole can better eliminate Helicobacter pylori, reduce the expression of COX-2 and other molecules, and play a better clinical effect.

## Figures and Tables

**Figure 1:** Improvement time of clinical symptoms of the two groups of patients: (a) improvement time of belch: the improvement time of belching in the OG was shorter than that in the CG (*p* < 0.05); (b) improvement time of epigastric pain: the improvement time of epigastric pain in the OG was shorter than that in the CG (*p* < 0.05); (c) improvement time of acid reflux: the improvement time of acid reflux in the OG was shorter than that in the CG (*p* < 0.05); (d) improvement time of abdominal distension: the improvement time of abdominal distension in the OG was shorter than that in the CG (*p* < 0.05). ∗ means compared with the CG, *p* < 0.05.

The article "Clinical Effect of Clarithromycin Combined with Tinidazole on Helicobacter pylori-Related Gastritis and Its Influence on COX-2 Expression" was retracted in 2024. Reasons: signs of a paper mill; suspected computer-generated content; unreliable results or conclusions; concerns about the data.

**Figure 2:** Relative expression levels of COX-2 and Bcl-2 in the two groups: (a) COX-2 mRNA: after treatment for 14 d and 30 d, COX-2 mRNA levels in the two groups decreased evidently, and Cox-2 mRNA levels in the OG were lower than those in the CG after treatment for 14 d (*p* < 0.05), but there was no difference between the two groups after treatment for 30 d (*p* > 0.05); (b) COX-2 protein: after 14 days and 30 days of treatment, the COX-2 protein level in the OG was evidently lower than that in the CG (*p* < 0.05), but there was no difference between the CG and the OG after 30 days of treatment (*p* > 0.05); (c) Bcl-2 mRNA: after treatment for 14 d and 30 d, the Bcl-2 mRNA level in the OG was evidently lower than that in the CG (*p* < 0.05), but there was no difference between the CG and the OG after treatment for 30 d (*p* > 0.05); (d) Bcl-2 protein: after 14 days and 30 days of treatment, the protein level of Bcl-2 in the OG was evidently lower than that in the CG (*p* < 0.05), but there was no difference between the CG and the OG after 30 days of treatment (*p* > 0.05). ∗ means compared with before treatment, *p* < 0.05; ∗∗ means compared with 14 days after treatment, *p* < 0.05.

**Figure 3:** Levels of inflammatory factors in the two groups: (a) IL-1: after 14 days and 30 days of treatment, IL-1 levels in the two groups decreased evidently, IL-1 levels in the OG were lower than those in the CG after 14 days of treatment (*p* < 0.05), but there was no difference between the two groups after 30 days of treatment (*p* > 0.05); (b) IL-4: after 14 days and 30 days of treatment, the levels of IL-4 in the OG were evidently lower than those in the CG (*p* < 0.05), but there was no difference between the CG and the OG after 30 days of treatment (*p* > 0.05); (c) CRP: after 14 days and 30 days of treatment, the levels of CRP in the OG were evidently lower than those in the CG (*p* < 0.05), but there was no difference between the CG and the OG after 30 days of treatment (*p* > 0.05). ∗ means compared with before treatment, *p* < 0.05; ∗∗ means compared with 14 days after treatment, *p* < 0.05.

**Figure 4:** Nutritional index levels of patients in the two groups: (a) ALB: after treatment for 14 d and 30 d, the ALB levels of patients in the two groups increased evidently, and the ALB levels in the OG were lower than those in the CG after treatment for 14 d and 30 d (*p* < 0.05); (b) Tf: after 14 days and 30 days of treatment, the Tf level in the OG was evidently higher than that in the CG (*p* < 0.05); (c) PA: after treatment for 14 days and 30 days, the PA level in the OG was evidently higher than that in the CG (*p* < 0.05). ∗ means compared with before treatment, *p* < 0.05; ∗∗ means compared with 14 days after treatment, *p* < 0.05.

The article "Clinical Effect of Clarithromycin Combined with Tinidazole on Helicobacter pylori-Related Gastritis and Its Influence on COX-2 Expression" was retracted in 2024. Reasons: signs of a paper mill; suspected computer-generated content; unreliable results or conclusions; concerns about the data.

**Table 1:** Related primers.

Factor	Upstream primer	Downstream primer
COX-2	5′-TGAAACCCACTCCAAACACAG-3′	5′-TCATCAGGCACAGGAGGAAG-3′
Bcl-2	5′-TGGGATGCCTTTGTGGAACTAT-3′	5′-AGAGACAGCCAGGAGAAATCAAAC-3′
GAPDH	5′-TGCGAGTACTCAACACCAACA-3′	5′-GCATATCTTCGGCCCACA-3′

**Table 2:** General data.

Group	OG (*n* = 80)	CG (*n* = 50)	*t*/*X*^2^	*p*
Gender			0.06	0.802
Male	43 (55.00)	28 (56.00)		
Female	37 (45.00)	22 (43.00)		
Average age (years)	42.13 ± 1.21	41.87 ± 1.53	1.08	0.284
BMI (kg/m^2^)	26.82 ± 2.75	27.17 ± 2.93	0.69	0.493
Years of education	10.23 ± 1.47	9.97 ± 1.69	0.93	0.356
Patient's family residence			0.31	0.575
Rural	36 (45.00)	20 (40.00)		
Urban	44 (55.00)	30 (60.00)		
Patient's family type			0.07	0.785
Other	16 (20.00)	11 (22.00)		
Core family	64 (80.00)	39 (78.00)		
Drinking			0.81	0.367
Yes	66 (82.50)	38 (76.00)		
No	14 (17.50)	12 (24.00)		
History of hypertension				
Yes	52 (77.50)	41 (82.00)		
No	28 (22.50)	9 (18.00)		
History of hyperlipidemia			0.01	0.952
Yes	62 (77.50)	41 (82.00)		
No	18 (22.50)	9 (18.00)		
History of diabetes			0.09	0.759
Yes	58 (72.50)	35 (70.00)		
No	22 (27.50)	15 (30.00)		

**Table 3:** Total effective rate.

Classification	OG (*n* = 80)	CG (*n* = 50)	*X* ^2^	*p*
Number of reinfection cases	4 (5.00)	7 (14.00)	—	—
Number of uncleared cases	2 (2.50)	5 (10.00)	—	—
Number of cleared cases	74 (92.50)	38 (76.00)	—	—
Clearance rate (%)	76 (92.50)	38 (76.00)	7.02	0.008

**Table 4:** Total effective rate.

Classification	OG (*n* = 80)	CG (*n* = 50)	*X* ^2^	*p*
Cured	34 (42.50)	17 (34.00)	—	—
Markedly effective	44 (55.00)	15 (30.00)		
Effective	20 (25.00)	11 (22.00)	—	—
Ineffective	2 (2.50)	7 (14.00)	—	—
Total effective rate (%)	78 (97.50)	43 (86.00)	6.32	0.012

**Table 5:** Incidence of complications.

Classification	OG (*n* = 80)	CG (*n* = 50)	*X* ^2^	*p*
Nausea	1 (1.25)	5 (10.00)	—	—
Dizzy	3 (3.75)	4 (8.00)	—	—
Vomiting	1 (1.25)	1 (2.00)	—	—
Incidence of adverse reactions (%)	5 (6.25)	10 (20.00)	5.70	0.017

## Data Availability

The authors confirm that the data supporting the findings of this study are available within the article.
